The article "Oncogenic extracellular HSP70 disrupts the gap-junctional coupling between capillary cells" was retracted in 2025. Reasons: duplicated images; original data or images not available.

# Oncogenic extracellular HSP70 disrupts the gap-junctional coupling between capillary cells

**DOI:** 10.18632/oncotarget.3522

**Published:** 2015-03-10

**Authors:** Dominique Thuringer, Kevin Berthenet, Laurent Cronier, Gaetan Jego, Eric Solary, Carmen Garrido

**Affiliations:** ^1^ INSERM, U866, Faculty of Medecine, Dijon, France; ^2^ CNRS ERL7368, STIM Lab, University of Poitiers, Poitiers, France; ^3^ University of Burgundy, Dijon, France; ^4^ INSERM, U1009, Institut Gustave Roussy, Villejuif, France; ^5^ CGFL, BP77980 21000 Dijon, France

**Keywords:** HSP, Cx43, pannexin, Ca^2+^ oscillations, ATP release

## Abstract

High levels of circulating heat shock protein 70 (HSP70) are detected in many cancers. In order to explore the effects of extracellular HSP70 on human microvascular endothelial cells (HMEC), we initially used gap-FRAP technique. Extracellular human HSP70 (rhHSP70), but not rhHSP27, blocks the gap-junction intercellular communication (GJIC) between HMEC, disrupts the structural integrity of HMEC junction plaques, and decreases connexin43 (Cx43) expression, which correlates with the phosphorylation of Cx43 serine residues. Further exploration of these effects identified a rapid transactivation of the Epidermal Growth Factor Receptor in a Toll-Like Receptor 4-dependent manner, preceding its internalization. In turn, cytosolic Ca^2+^ oscillations are generated. Both GJIC blockade and Ca^2+^ mobilization partially depend on ATP release through Cx43 and pannexin (Panx-1) channels, as demonstrated by blocking activity or expression of channels, and inactivating extracellular ATP. By monitoring dye-spreading into adjacent cells, we show that HSP70 released from human monocytes in response to macrophage colony-stimulating factor, prevents the formation of GJIC between monocytes and HMEC. Therapeutic manipulation of this pathway could be of interest in inflammatory and tumor growth.

## INTRODUCTION

Heat shock protein 70 (HSP70) which was initially described as an intracellular protein [1-3] is also released into the circulation under various stress conditions [4-9]. Circulating HSP70 is increased in pathological conditions including cancer cell invasiveness and metastasis [10-12]. Irrespective of whether HSP70 enters the circulation via an active or passive release mechanism, the role of this extracellular HSP70 remains poorly understood.

High levels of circulating HSP70 are reported to correlate with monocyte adhesion to endothelial cells [13]. Among the systems that mediate cell-to-cell interaction, gap junctional intercellular communication (GJIC) is an important modulatory factor for growth, migration and differentiation of cells. Gap junctions are plasma membrane domains containing intercellular channels that allow a direct exchange of ions and small molecules between adjacent cells. The channels are composed of two hemichannels and are formed when a hemichannel from one cell docks with a symmetrically opposed hemichannel from a neighboring cell [14]. Each hemichannel is an oligomer of six proteins named connexins (Cx), which form the central pore of the channel. Connexins expressed within the vasculature include Cx37, 40, 43 and 45 [15, 16]. Although they are differentially expressed along the vascular tree, Cx43 is the most widely and highly expressed protein in all cell models and human tissues. The permeability of gap junctions can be affected by a number of mechanisms, including changes in cytosolic ion concentrations and Cx43 phosphorylation [17]. Their aberrant function has been associated with a number of pathological conditions, including cancer and inflammation [18-21].

The article "Oncogenic extracellular HSP70 disrupts the gap-junctional coupling between capillary cells" was retracted in 2025. Reasons: duplicated images; original data or images not available.

Whereas the role of Cx hemichannels formed by Cx43 in modulation of monocytes-endothelial adhesion is well identified [22, 23], the role of the paracrine intercellular communication is less clear. This paracrine communication does not require cell-cell apposition, as it involves release of one or more signalling molecules into the extracellular medium, and their subsequent interaction with receptors, such as G protein-coupled receptors (GPCRs), on neighboring cells [24]. One of these paracrine factors is adenosine triphosphate (ATP), which is released through unpaired Cx hemichannels (not connecting cells) and propagates intercellular Ca^2+^ waves.

Extracellular HSP70 induces signal transduction through the LPS receptor CD14 in monocytes and macrophages [25, 26]. In malignant cells, HSP70 also induces a TLR4-dependent EGFR phosphorylation, which triggers MAPK signaling [6, 25, 27]. Because LPS or EGF induce Cx43 phosphorylation leading to GJIC abrogation [28, 29], we examined whether extracellular HSP70, exogenously added or released from circulating monocytes, modulates GJIC and Cx43-hemichannel functions in human microvascular endothelial cells (HMEC) via the engagement of specific membrane receptor-associated signaling pathways in HMEC.

## RESULTS

### Extracellular recombinant human HSP70 (rhHSP70) blocks the gap junction intercellular communication (GJIC) between human microvascular endothelial cells (HMEC)

The effects of rhHSP70 were analyzed on the functionality of gap junctions established between HMEC in confluent monolayer by using the gap-FRAP technique [30, 35]. Briefly, HMEC were loaded with a diffusible tracer (calcein/AM), and the fluorescence of investigated cells was suppressed by a laser beam. The recovery of fluorescence in these cells, which results from the intercellular diffusion of calcein from neighboring cells, was recorded to measure the diffusion rate constant k (min^−1^), an index of gap junction permeability. Fig. 1A shows typical changes in the fluorescence of cells, before and after photobleaching. rhHSP70 was used at 5 μg/ml (Fig. 1B, open circles), a concentration that evoked both maximal spreading of HMEC spheroids (Suppl. Fig. S1) and increase in cell motility (Suppl. Fig. S2). rhHSP70 prevented the fluorescence recovery normally observed in cells exposed to control solution (black circles), demonstrating that rhHSP70 blocked the GJIC between HMEC (Fig. 1B). A time-dependent decrease in k was observed within 1 h (from 0.417 ± 0.100 min^−1^ in untreated to 0.032 ± 0.014 min^−1^ in rhHSP70-treated cells; mean ± SD, n=8; Fig. 1C). In comparison, HMEC exposure to rhHSP27 rather increased k (from 0.488 ± 0.207 min^−1^ in untreated cells to 0.643 ± 0.277 min^−1^; n=8). Addition of polymyxin B (PMB100 ng/ml) did not prevent the time-dependent decrease in k value observed with rhHSP70 (from 0.445 ± 0.111 min^−1^ in control to 0.097 ± 0.100 min^−1^; n=3). Thus, the rhHSP70-induced GJIC inhibition is mainly caused by the rhHSP70 protein itself, rather than by any contaminating endotoxin.

The article "Oncogenic extracellular HSP70 disrupts the gap-junctional coupling between capillary cells" was retracted in 2025. Reasons: duplicated images; original data or images not available.

**Fig 1:** Extracellular rhHSP70 inhibits the endothelial gap-junction coupling A. FRAP analysis of cell-to-cell communication. Digital images of fluorescence distribution in a HMEC monolayer at three times during a typical gap-FRAP experiment: prebleach, just after bleaching (0 min) and after fluorescence recovery (8 min). Polygons 2-5 are bleached cells, and polygon 1 is an unbleached control cell used for correction of the artefactual loss of fluorescence. Bars 20 μm. Corresponding fluorescence intensities (% of prebleach value) versus time in tested cells. Note the fluorescence recovery follows an exponential time course when the bleached cells are interconnected by open gap-junction channels to unbleached cells (polygons 2-5). The relative permeability of gaps is given by the time constant k. B. Graph represents mean ± SEM of the fluorescence redistribution after photobleaching in coupled HMEC in control (●) or after 60 min (○) with rhHSP70 (5 μg/ml). (C) Histogram shows k values measured after rhHSP70 addition for 0, 30, 60 min and 24 h (mean ± SD, n=8; **P<0.01, *P<0.05 *vs* control [t=0 min]).

### Extracellular rhHSP70 modulates Cx43 protein expression and phosphorylation

Connexin 43 (Cx43) which is the most widely and highly expressed gap junction protein [36], is detected at the level of gap junction plaques and within the intracellular space of HMEC cultures (Fig. 2A). Consistent with GJIC abrogation, rhHSP70 decreased Cx43 at the plasma membrane within 30 min and disrupted the Cx43 gap junction plaques within 1h. As Cx43 incorporated into gap junction plaques is insoluble in Triton X-100 [32], we subjected HMEC to a Triton X-100 fractionation assay and determined the relative amount of Cx43 in the junctional plaques. Fig. 2B shows that rhHSP70 provoked a drastic reduction in Cx43 expression at the plasma membrane (46 ± 6% of control after 1 h; **P<0.001, n=5). We did not detect significant changes in expression of the other endothelial-specific Cx37 and Cx40 (Suppl. Fig. S3).

The article "Oncogenic extracellular HSP70 disrupts the gap-junctional coupling between capillary cells" was retracted in 2025. Reasons: duplicated images; original data or images not available.

Specific serine phosphorylations in the C-terminal tail of Cx43 [37] were increased by rhHSP70 within 1 h (Fig. 2C), as expected for a blockage of GJIC [38, 39]. All these phosphorylating effects of rhHSP70 were antagonized by cell pretreatment with a neutralizing antibody against toll-like receptors (TLR) 4 (*Ab*TLR4) (Fig. 2D).

Zonula occludens 1 (ZO-1) is the major protein that interacts with Cx43, precisely through its C-terminal region, to form functional gap junction plaques [40, 41]. Interestingly, inhibition of ZO-1/Cx43 interaction has been shown to promote Cx43 phosphorylation on Ser368. As shown in Fig. 2E, HMEC displayed large cell border-localized ZO-1 which was not delocalized upon 1 h of rhHSP70 application. Furthermore ZO-1 coimmunoprecipitated with Cx43 in control as well after 30 min of cell exposure to rhHSP70 but not in the following time periods (Fig. 2F). Disruption of the Cx43/ZO-1 interaction coincides not only with the reduction of Cx43 present at the plasma membrane, but also its phosphorylation at Ser368, as previously reported [42] (but not of Tyr265, Suppl. Fig. S3).

**Fig 2:** Extracellular rhHSP70 modules membrane level and phosphorylation of Cx43 A. Immunofluorescence detection of Cx43 (green) in HMEC after treatment with 5μg/ml rhHSP70 for indicated times (DAPI staining of nuclei). Arrows indicate Cx43 plaques. Representative of 5 experiments. Bar 20 μm. B. Western blot of the total and membrane fraction (Triton X-100 insoluble) of Cx43. P0, P1 and P2 denotes the three major Cx43 migration bands. Cell membrane lysates immunoblotted for Cx43, after treatment with rhHSP70 for time periods as indicated (Hsc70 as loading control). Right panel shows changes in band intensity of the membrane fraction related to the total Cx43 expression level (mean ± SD, n=5; **P<0.01, *P<0.05 *vs* control [t=0 min] in all cases). C. Effect of rhHSP70 on Cx43 phosphorylation pattern. Western blots using three different antibodies against the carboxy terminal part of Cx43 to detect phosphorylation on serine at position Ser262, Ser255 and Ser368 (representative of 5 experiments). D. rhHSP70 leads to phosphorylate Cx43 in a TLR4-dependent manner. Western blot showing phosphorylation on Ser368. When indicated, cells were pre-treated for 60 min with polymyxin B (PMB10 μM) or the neutralysing anti-TLR4 (*Ab*TLR4 10 μg/ml). rhHSP70 was (or not) added for 60 min (representative of 5 experiments). Histogram shows changes in the phosphorylated status of Cx43 in response to 60 min of cell treatment with rhHSP70 (black) or rhHSP70 plus AbTLR4 (grey), expressed as percentage of control (mean ± SD, n=5; **P<0.01, *P<0.05 *vs* control). E. Immunofluorescence detection of ZO-1 in HMEC after exposure to rhHSP70 for indicated times. Representative of 5 experiments. Cell nuclei stained with DAPI. Bar 20 μm. F. Coimmunoprecipitation of Cx43 and ZO-1 in HMEC, stimulated or not by rhHSP70 for time periods as indicated. The total Cx43 shows slight variations in the unphosphorylated form P0 and the phosphorylated forms P1 and P2 (Hsc70 as loading control; representative of 4 experiments).

The article "Oncogenic extracellular HSP70 disrupts the gap-junctional coupling between capillary cells" was retracted in 2025. Reasons: duplicated images; original data or images not available.

### Extracellular rhHSP70 mediates EGFR transactivation contributing to GJIC abrogation

Heat shock and exogenous HSP70 were shown to activate toll-like receptors (TLR) 2 and 4, as well as to promote their association with the epidermal growth factor receptor (EGFR) and the receptor phosphorylation [6]. Since TLR2 is not detected in HMEC, we hypothesized that rhHSP70 may transactivate EGFR through its interaction with TLR4. Accordingly, the rhHSP70-induced EGFR phosphorylation was prevented by the neutralizing *Ab*TLR4 antibody while being unaffected by PMB (Fig. 3A).

After boiling rhHSP70 solution for 30 min, which denaturizes the protein but not LPS, EGFR phosphorylation was no longer observed, indicating that the effect of intact rhHSP70 was due to HSP70 itself (Fig. 3B) and there was no active endotoxin in solutions. Pre-treatment of HMEC with AG490 (50μM), a kinase inhibitor of JAK2 and EGFR, partially prevented EGFR phosphorylation (by 45%; n=6; P<0.01).

By adding an HA motif at its N-terminus, we produced a tagged rhHSP70 that was used to distinguish the exogenous from the endogenous proteins. The purified rhHSP70-HA molecule was a single 70-kDa protein as much functional as the commercially available recombinant molecule (Suppl. Fig. S4). rhHSP70-HA was observed to be internalized into serum-starved HMEC within 5 minutes, and to partially co-localize with EGFR (Fig. 3C).

The AKT activation, which is crucial to disrupt GJIC by causing phosphorylation of Ser368 in Cx43 [43, 44], was rapidly induced by rhHSP70 (within 5 min) in a TLR4-dependent manner (Fig. 3D). The EGFR tyrosine kinase inhibitor, gefitinib (10μM) also antagonized the inhibitory effect of rhHSP70 on GJIC (Fig. 3E). Altogether, our data suggest that rhHSP70 transactivates EGFR.

The article "Oncogenic extracellular HSP70 disrupts the gap-junctional coupling between capillary cells" was retracted in 2025. Reasons: duplicated images; original data or images not available.

**Fig 3:** Extracellular rhHSP70 induces a TLR4-dependent EGFR transactivation leading to the GJIC abrogation A. Western blot analysis of EGFR Tyr-1068 phosphorylation and TLR4 expression in HMEC, unstimulated (control) or stimulated with rhHSP70 or LPS (1 μg/ml) for 15 min. When indicated, cells were pre-treated for 60 min with polymyxin B (PMB10 μM) or the neutralysing anti-TLR4 (*Ab*TLR4 10 μg/ml). Lower panel shows changes in the band intensity (mean ± SD, n=3; Hsc70 as loading control). B. Tyrosine phosphorylation of EGFR by rhHSP70 involves the kinase JAK2. Western blot analysis of EGFR phosphotyrosine (P-Tyr) after EGFR immunoprecipitation in HMEC. Cell pretreatment with the kinase inhibitors AG1478 (AG14; 5μM), CGP77675 (CGP; 1μM), AG490 (50μM) for 30 min before exposure to rhHSP70 or 100 ng/ml EGF for 15 min. A boiled rhHSP70 (100°C, 30 min) known to denaturize protein but not LPS, was used to evaluate the contribution of contaminants to the EGFR activation. Lower panel shows changes in band intensity (mean ± SD, n=5; **P<0.01, *P<0.05 *vs* rhHSP70 [t = 0 min] with AG490). C. *P*artial co-localization of rhHSP70 and EGFR. HMEC were stimulated with rhHSP70-HA for 5 min and double-stained for EGFR (ErbB1). Representative micrographs and corresponding cross-sections (xz and yz) showing a three-dimensional stack of rhHSP70 (green), EGFR (red) and the combined image of co-localization (yellow); DAPI staining of nuclei. Optical section of 0.5 μm thickness (n=3, bar 20 μm). D. Phosphorylation of AKT. Cells were exposed to rhHSP70 for the indicated time periods, and lysates were immunoblotted using antibodies recognizing phosphorylated or total forms of AKT. When indicated, cells were pretreated for 60 min with the neutralysing anti-TLR4 (*Ab*TLR4 10 μg/ml). Lower panel shows corresponding changes in the band intensity. E. Contribution of EGFR signaling to rhHSP70-induced GJIC inhibition. Diffusion rate constants k determined from recovery curves for HMEC after 1 h in control, Gefitinib (Gefi; 10μM) or Gefi plus rhHSP70 (mean ± SD, n=4; **P<0.01, *P<0.05 vs control).

### Extracellular rhHSP70 induces intracellular Ca^2+^ mobilization

Since EGFR engagement activates a calcium-dependent signaling [45, 46], we measured the 340/380 nm ratio of fura-2 fluorescence, reflecting the cytosolic [Ca^2+^]i in PM-pretreated, fura-2-loaded HMEC (Fig. 4A, upper trace). In nominally Ca^2+^-free bath conditions, rhHSP70 induced a transient increase in [Ca^2+^]i within 1–3 min, which was followed by three or more Ca^2+^ waves. These oscillations, never spontaneously observed in control (middle trace), could be prevented by the selective inhibitor of endoplasmic reticulum Ca^2+^-ATPase, thapsigargin (4μM), suggesting that rhHSP70 recruits Ca^2+^ from intracellular stores (lower trace). Furthermore, rhHSP70 induced phosphorylation of AKT, ERK and SAPK/JNK within 5–10 min, which was significantly attenuated by the Ca^2+^ chelator BAPTA/AM (Suppl. Fig. S5).

The article "Oncogenic extracellular HSP70 disrupts the gap-junctional coupling between capillary cells" was retracted in 2025. Reasons: duplicated images; original data or images not available.

The EGFR tyrosine kinase inhibitor, gefitinib (10 μM), attenuated the Ca^2+^ signal elicited by rhHSP70, i.e. the initial peak amplitude was decreased at 56 ± 3% of the control amplitude (n=20; P<0.05; Fig. 4B). These results demonstrate that an amplification loop involving intracellular calcium and EGFR activation mediates the effects of rhHSP70 in HMEC.

EGFR transactivation is known to stimulate phospholipase C (PLC), leading to inositol 1,4,5-trisphosphate (InsP3) formation and release of Ca^2+^ from InsP3-sensitive Ca^2+^-stores. The extracellular application of U-73122 (5 μM), an inhibitor of PLC, reduced both the number and amplitude of rhHSP70-evoked Ca^2+^ oscillations (Fig. 4C) [47]. In contrast, the same dose of its inactive analog, U-73343, had no effect. Furthermore, the cell pretreatment with BTP-2 (20 μM), a cell-permeable blocker of store-operated Ca^2+^ entry (SOCE), decreased both frequency and amplitude of Ca^2+^ oscillations without affecting the initial peak of Ca^2+^ release and the basal [Ca^2+^]i (Fig. 4D). Pretreatment with 2-APB (50 μM), a blocker of InsP3 receptors [48], decreased basal [Ca^2+^]i and suppressed Ca^2+^ oscillations. Thus, intracellular Ca^2+^ oscillations evoked by rhHSP70 are related to the initial release of Ca^2+^ from InsP3-sensitive intracellular Ca^2+^-stores.

**Fig 4:** Extracellular rhHSP70 induces intracellular Ca^2+^ mobilization A. rhHSP70 induced Ca^2+^ release from internal stores in HMEC. Data are expressed as the 340/380 nm excitation ratio in one cell to observe oscillations in [Ca^2+^]i because the oscillatory process is not synchronized in cells of the same monolayer. External additions of drugs are indicated by arrows. Changes in external calcium bath conditions are indicated on the bottom of traces. In most cases, drugs were initially applied in the absence (0 Ca) then in Ca^2+^ (1.8 mM) containing solution to reveal Ca^2+^ release from internal stores then external Ca^2+^ entry, respectively (representative from 50 cells; n=10). No calcium increase was induced by the cell superfusion of the control bath solution (middle trace) while thapsigargin (TSG 4μM) always produced a drastic increase in [Ca^2+^]i (lower trace; Representative from 50 cells; n=4). B. Contribution of EGFR to rhHSP70-induced Ca^2+^ signaling. Superimposed traces from cells preincubated with the EGFR (ErbB1) inhibitor, gefitinib (10 μM for 30 min; in red), before the addition of rhHSP70 (Representative from 50 cells; n=5). C. Effects of phospholipase C (PLC) inhibitor U-73122 (5 μM) and its inactive analog U-73343 (5 μM) on the rhHSP70-induced Ca^2+^ oscillations. Drugs were applied without (0 Ca) then with extracellular Ca^2+^ (1.8 mM) (representative from 50 cells; n=5). D. Ca^2+^ oscillations required both Ca^2+^ release from internal stores and store operated Ca^2+^ entry (SOCE). Cells were pretreated with the selective SOCE inhibitor, BTP-2 (20 μM; 20 min), before challenged with rhHSP70 (Representative from 30 cells; n=4).

The article "Oncogenic extracellular HSP70 disrupts the gap-junctional coupling between capillary cells" was retracted in 2025. Reasons: duplicated images; original data or images not available.

### Ca^2+^ mobilization and GJIC blockage are partially dependent on ATP release by HMEC

Extracellular ATP inactivation with apyrase (20 U/ml) significantly reduced both the frequency and amplitude of [Ca^2+^]i oscillations while keeping fairly conserved the amplitude of the initial Ca^2+^ peak (Fig. 5A). Moreover, apyrase partially antagonized the blocking action of rhHSP70 on GJIC (Fig. 5B). Cell exposure to rhHSP70 induced a significant release of ATP as demonstrated using the luciferin-luciferase bioluminescence assay (Fig. 5C).

Given that rhHSP70-induced cytosolic Ca^2+^ oscillations in HMEC depend, at least in part, on the release of ATP and subsequent P2 purinergic receptor activation, we supposed that Cx43 hemichannels could act as a putative pathway of ATP release. Inhibition of Cx43 channels, either with 18βGA (10 μM, n=2; not shown) or with the mimetic peptide Gap26 (500 μM) totally suppressed the rhHSP70-induced ATP release from HMEC (Fig. 5C) and significantly attenuated rhHSP70-induced Ca^2+^ response, especially the oscillatory process (Fig. 5D). The remaining ATP release, also observed in control cells, was unable to evoke Ca^2+^ oscillations in HMEC (Fig. 5D) and could be blocked by the vesicular transport inhibitor brefeldin A (20 μM; not shown).

Recent evidence emerged indicating that a cross-inhibition of pannexin (Panx) channels, especially Panx-1, by mimetic peptides (Gap26) and carbenoxolone, is involved in ATP release and Ca^2+^ currents in various cell types [49]. Therefore we tested a specific inhibitor of Panx-1, probenecid (Prb), at a dose that does not affect Cx channels [50]. Prb reduced rhHSP70-evoked Ca^2+^ oscillations without affecting the initial peak (Fig. 5E) and totally blocked the rhHSP70-evoked ATP (Fig. 5F). The total inhibition of cytosolic Ca^2+^ oscillations was achieved with Gap26. When the Cx43 expression was reduced by siRNA (Fig. 5F), the rhHSP70-induced ATP release was significantly decreased (by 40%), and further abolished by Prb (Fig. 5F).

The article "Oncogenic extracellular HSP70 disrupts the gap-junctional coupling between capillary cells" was retracted in 2025. Reasons: duplicated images; original data or images not available.

**Fig 5:** The rhHSP70-induced ATP release contributes to endothelial Ca^2+^ oscillations A. Contribution of the ATP release to the rhHSP70-evoked Ca^2+^ oscillations in HMEC. Cells were either untreated (black) or pretreated for 30 min with 20 U/ml apyrase (red) before to be exposed for 60 min to rhHSP70 (representative of 20 cells; n=5). B. Apyrase partially antagonizes the inhibitory effect of rhHSP70 on the GJIC between HMEC pretreated by apyrase then apyrase plus rhHSP27. Histogram shows the diffusion k constant measured after 60 min of cell treatments (mean ± SD, n=4; *P*-values<0.05 *vs* control). C. rhHSP70-induced ATP release from HMEC is blocked by Gap26 (500 μM). Extracellular ATP was measured by Luciferase assay (means ± S.D., n=3, *P*-values<0.05 *vs* control). D. Contribution of Gap26-sensitive channels to the rhHSP70-induced Ca^2+^ oscillations. Cells pretreated with *Gap26* (500 μM for 30 min; red) before rhHSP70 (representative of 20 cells; n=5). E. Pannexin-1 modulates the Ca^2+^ oscillatory response to rhHSP70. Superimposed traces obtained from cells stimulated with rhHSP70 in the presence or absence of the Panx-1 blocker, 100 μM probecenid (Prb; green), or Prb plus Gap26 (red) (Representative of 10 cells; n=5). F. siRNA Cx43 knockdown attenuates the rhHSP70-induced ATP release. HMEC were transfected with Cx43 and control siRNA 48 h prior to various analyses. Insert is representative western blot showing the specific depletion of Cx43. Histogram shows the amounts of ATP released (relative to control cells) in response to rhHSP70 (1h). In some cases, transfected cells were exposed to 100 μM Prb (mean values ± SD, n=5; **P<0.01, *P<0.05 vs control).

### HSP70 release from stimulated human monocytes prevents heterocellular GJIC with HMEC

The release of ATP and subsequent activation of endothelial intracellular Ca^2+^ signalling are reported to modulate monocyte adhesion to endothelial cells and their transendothelium migration [23, 51]. Exposure of human, peripheral blood monocytes to M-CSF for 12 hours increased the expression and release of HSP70, without affecting Cx43 expression and phosphorylation (Fig. 6A, B, C). The amount of HSP70 secreted by monocytes seems very low compared with the exogenously added in HMEC cultures. However this was a dosage for the whole fluid bathing the cells whereas the secretion by monocytes must be considered in their closed vicinity near the endothelial cell. So the real quantity of HSP70 secreted by the monocyte and collected by the endothelial cell is certainly much higher that the dose measured (diluted) in the whole bath. Knocking down HSP70 with a specific *si*RNA reduced by about 80% the amount of HSP70 found after 12 h into the bath of M-CSF-treated monocytes (Fig. 6D). M-CSF-stimulated monocytes increased ATP release by HMEC, which could be mediated by HSP70 released from these monocytes (Fig. 6E).

The article "Oncogenic extracellular HSP70 disrupts the gap-junctional coupling between capillary cells" was retracted in 2025. Reasons: duplicated images; original data or images not available.

**Fig 6:** The HSP70 release by monocytes alters their coupling with HMEC A. M-CSF (100 nM) increases HSP70 expression in monocytes (representative of 5 experiments; Hsc70 as loading control). B. Cx43 expression in monocytes is not affected by 12h-treatment with M-CSF or rhHSP70 (representative of 3 experiments). C. M-CSF induced HSP70 release. Amounts of HSP70 measured by ELISA in supernatant of monocytes untreated (control) or treated with 100 nM M-CSF for 12 h (mean ± SD; n=4; **P-values <0.01). D. siRNA HSP70 knockdown. Cultured monocytes were transfected with HSP70 or control siRNA 48h prior to various analysis. Left, western blot analysis of protein extracts from cells treated with M-CSF for 12 h. Right, histogram shows HSP70 release by transfected monocytes in response to 100 nM M-CSF for 12 h (mean ± S.D., n=4; representative of 4 experiments). E. The ATP release by HMEC/monocyte cocultures is mainly due to HMEC (bioluminescence assay; means ± S.D. n=3; **P-values<0.01, *P-values<0.05 vs control). F. Functional GJIC between monocytes and HMEC. Monocytes (donors) were preloaded with calcein/AM and DiL-C18. Calcein diffuses through gap junctions, while DiL-C18 does not. Labelled monocytes are then plated with unlabeled HMEC monolayer (receivers). HMEC establishing GJIC with monocytes become fluorescent by calcein diffusion. Only siRNA HSP70-transfected monocytes establish GJIC with HMEC and exogenously added rhHSP70 (5μg/ml) improved it. Phase-contrast microphotographs after 3 h of culture (representative of 6 experiments; Bar 100 μm).

To evaluate the impact of released HSP70 on the establishment of GJIC between monocytes and HMEC, these monocytes were double loaded with calcein, a dye that is able to pass through gap junctions, and with DiL, a membrane-bound stain used to distinguish cell donor (monocyte) from recipient cells (HMEC) (Fig. 6F). Note that calcein is an intracellular dye that becomes fluorescent after hydrolysis by cytosolic esterases [52]. After hydrolysis, calcein is highly charged and therefore impermeable to cell membranes; it is thought to travel from cell to cell through gap junctions [35, 53]. DiL, conversely, does not travel from cell to cell [54]. Preloaded monocytes were then plated with unlabeled HMEC monolayer. After 3 hours of co-culture, unstimulated monocytes remained in suspension, whereas M-CSF-treated cells adhered to the endothelial monolayer (Fig. 6F). The HSP70 knock-down by using a specific *si*RNA, promoted calcein transfer from monocyte to endothelial cells, attesting formation of GJIC. The supplementary addition of rhHSP70 to the bath reversed it. The gap-junction blockers, carbenoxolone (200 μM) and 18βGA (500 μM) similarly blocked this heterocellular dye transfer (not shown). These results make clear that released HSP70 prevents cell-to-cell communication between monocytes and HMEC.

The article "Oncogenic extracellular HSP70 disrupts the gap-junctional coupling between capillary cells" was retracted in 2025. Reasons: duplicated images; original data or images not available.

Dye coupling was also seen with the non-transfected monocytes pretreated by the adenosine derived inhibitor of HSP70, VER155008 (Fig. 7A), i.e. VER155008-treated cells established functional gap junctions with HMEC in response to M-CSF. VER155008 treatment did not change the high level of HSP70 protein expressed in cells stimulated by M-CSF (Fig. 7B). Treatment of HMEC alone by VER155008 improved the blocking action of rhHSP70 on GJIC (Fig. 7C).

To explore the role of Cx43 in monocyte-endothelial cell interactions, HMEC were transfected with siRNA Cx43 or control siRNA, and intercellular communication was tested 48 h later (Fig. 7D). Control HMEC cultures (transfected with control siRNA) showed extensive dye transfer of calcein from M-CSF-treated siRNA HSP70 monocytes (on average of 7 neighboring cells). The siRNA-mediated knockdown of Cx43 in endothelial cells did not affect the adhesion monocytes, but abolished (reduced by more 90% from control levels) the heterocellular GJIC. Upon stimulation by M-CSF, the transendothelial migration of monocytes in which HSP70 has been decreased by siRNA was strongly increased as compared to control cells (Fig. 7E). This “diapedesis” increase was abolished by knocking down the endothelial Cx43 expression.

**Fig 7:** The endothelial Cx43 expression is required for the transendothelial migration of monocytes A. The adenosine-derived inhibitor of HSP70, VER155008 (10 μM) favors the establishment of GJIC between monocytes (M-CSF stimulated) and HMEC within 3 h. Phase-contrast microphotographs are representative of 4 experiments. Bar 100 μm. Right, histogram represents the total cell number of HMEC receiving dye (calcein) per monocyte (mean ±SD, n=3; **P-values <0.01 vs control). B. VER155008 does not inhibit the HSP70 release by M-CSF-stimulated monocytes for 12 h (dosed by ELISA; mean ± SD, n=4; *P-values <0.05 vs control). C. VER155008 antagonizes the blocking effect of rhHSP70 on GJIC between HMEC (gap-FRAP analysis). Histogram shows the constant k measured for the coupled cells after 1 h of cell treatment (mean ± SD, n=4; *P-values<0.05 vs control). D. Effects of the endothelial Cx43 knockdown on the GJIC coupling between HMEC and HSP70 depleted monocytes. Cultured HMEC and monocytes were transfected respectively with siRNA Cx43 (HMEC) and siRNA HSP70 (monocytes) or control siRNA, 48h prior to various analysis. Insert is representative western blot showing the specific depletion of Cx43 in HMEC. Transfected monocytes (donors), stimulated overnight with M-CSF, were pre-loaded with calcein and DiL-C18 before to be plated. Microphotographs of monocytes in contact with transfected HMEC (receivers) after 3 h of culture (representative of 6 experiments; Bar 100 μm). Histogram represents the mean cell number of neighboring HMEC receiving dye (calcein) per monocyte (mean ±SD; n=50 labeled monocytes examined; n=3). E. Effects of the endothelial Cx43 knockdown and released HSP70 on the transendothelial migration of monocytes. Control or transfected HMEC monolayers grown on Transwells were kept in FCS-free conditions overnight. Control or transfected monocytes (3×10^5^) stimulated overnight by M-CSF, were labeled with phycoerythrin-conjugated anti-CD14+ before to be added into the wells. Cells migrating through the endothelial layers were counted (after 3 h). Data are percentage of total applied monocytes counted by flow cytometry (mean ± SD; n=5).

The article "Oncogenic extracellular HSP70 disrupts the gap-junctional coupling between capillary cells" was retracted in 2025. Reasons: duplicated images; original data or images not available.

## DISCUSSION

The major contribution of our study is the demonstration that extracellular HSP70, exogenously added or released from human circulating monocytes in response to M-CSF induction, activates a signaling cascade that decreases GJIC activity between HMEC and HMEC/monocytes reducing monocyte transmigration through the endothelium (Fig. 8). Thereby, HSP70 release may play a regulatory role in monocyte diapedesis when invading tissues to differentiate into macrophages or osteoclasts, depending on tissue microenvironment. Therapeutic manipulation of this pathway would be a strategy in various diseases such as chronic inflammatory diseases, osteoporosis, and cancer.

The protective functions of intracellular HSP70 are well documented whereas the role of extracellular HSP70 has been less explored [8, 11, 55]. Here, we show that extracellular HSP70 specifically decreases expression of Cx43 at the plasma membrane and induces hyper-phosphorylation of Cx43 in a time-dependent manner, leading to GJIC blockage. Since a reduced expression of Cx43 in endothelial cells has been shown to decrease the formation of vessels in Matrigel [19], this decreased expression may explain why rhHSP70 affects the spreading pattern of endothelial cells as compared to the typical sprouting when exposed to VEGF. The decreased expression of Cx43 in response to HSP70 is associated with the phosphorylation of its serine residues, which was shown to regulate gap junction channel formation, permeability, and turnover in other cell types [38]. In addition, rhHSP70 inhibits the ZO-1/Cx43 interaction at the plasma membrane, reducing the amount of Cx43 at the cell surface. Accordingly to Palatinus and coworkers [56], we confirm that inhibition of this interaction favors phosphorylation on Ser368. Specific phosphorylation of Cx43 has also been observed to promote GJIC inhibition in rat microvascular endothelial cells exposed to LPS [28].

The article "Oncogenic extracellular HSP70 disrupts the gap-junctional coupling between capillary cells" was retracted in 2025. Reasons: duplicated images; original data or images not available.

HSP70 was observed to physically interact with TLR4, which transactivates EGFR. Inhibition of TLR-4 and its downstream signaling cascade with specific neutralizing antibodies efficiently suppressed HSP70-induced tyrosine phosphorylation of EGFR in HMEC. The use of kinase inhibitors suggested that EGFR transactivation may only slightly depend on intrinsic EGFR tyrosine and Src kinase activities, but may require kinase activity that is partially inhibited by the tyrphostin AG490.

In several cell types including HMEC [57, 58], EGFR activation elicits an initial Ca^2+^ peak that depends on inositol-1,4,5-triphosphate (InsP3) through induction of Ca^2+^ release from intracellular stores, followed by a plateau phase dependent on a secondary Ca^2+^ entry from the extracellular compartment. The oscillatory behavior of secondary Ca^2+^ entry depends on the cell type. Extracellular HSP70 induces such a biphasic Ca^2+^ response in HMEC, *i.e*. an initial peak followed by [Ca^2+^]i oscillations in nominally Ca^2+^-free external conditions. As already described in EGF-treated cells [59], the source of Ca^2+^ responsible for these oscillations is the InsP3-sensitive endoplasmic reticulum (ER) store. Due to the modulation of InsP3 receptors by Ca^2+^, the “pacemarker” elevation which precedes the spikes could be explained by a slowly rising level of [Ca^2+^]i released by InsP3 until a threshold [Ca^2+^]i is reached to elicit the rapid upstroke [60, 61]. By using BTP-2, a blocker of store-operated Ca^2+^ entry (SOCE), and 2-APB, a potent blocker of InsP3 receptors, we show intracellular Ca^2+^ oscillations evoked by rhHSP70 are mainly due to the release of Ca^2+^ from InsP3-sensitive Ca^2+^-stores although the frequency of oscillations require calcium entry across the plasma membrane.

Release of ATP was shown to promote an oscillatory increase in cytosolic Ca^2+^ [62], underlying the paracrine intercellular communication [63-67]. Here we demonstrate that extracellular HSP70 leads to an immediate and robust release of ATP by HMEC. The Cx43 inhibition (Gap26) or knockdown only attenuated the ATP release from HSP70-treated HMEC, suggesting Cx43-hemichannels contribute but are not mainly involved in rhHSP70-induced ATP release. Note that a reduction of Cx43 expression not only lead to a reduction of gap junction function, but also might trigger more complex cellular alterations. In contrast, inhibition (Prb) of Panx-1 function or suppression of its expression (Suppl. Fig. S6) totally abolished rhHSP70-induced ATP release [49, 50, 68]. On the basis of inhibitor data and siRNA experiments, we conclude that Panx-1 channels mainly contribute to the observed rhHSP70-evoked ATP.

The article "Oncogenic extracellular HSP70 disrupts the gap-junctional coupling between capillary cells" was retracted in 2025. Reasons: duplicated images; original data or images not available.

Taken together, our experiments indicate that HSP70 released from M-CSF-treated monocytes does not affect monocyte adhesion to endothelial cells but prevents cell-cell communication between monocytes and HMEC. Note that Ca^2+^ chelation did not affect monocyte adhesion but slowed down monocyte transmigration through human microvascular endothelium [51]. The role of gap junctions in endothelial paracellular permeability is not well understood. Rather, adhesion complexes such as tight junctions and adherens junctions are established as regulators of permeability at the membrane, restricting paracellular flux [69]. From our observations, it is unlikely that the gap junctions contribute in adhesive function. Our studies also exclude a significant role of connexins as opening hemi-channels. Therefore, the connexins likely participate in the permeability response to inflammatory stimuli through their function in intercellular GJIC, by facilitating the intercellular exchange of signal that coordinate or enhance the response. In addition to Ca^2+^ ions, micro RNA may also pass through gap junctions, suggesting it as an additional candidate among signaling molecules [70]. Moreover, our data suggest that M-CSF, as secreted by endothelial cells in atherogenesis, contribute to the accumulation of monocytes at the site of inflammation by stimulating HSP70 release and subsequently inhibiting monocytes transmigration. Similar mechanisms could be involved in cancers where monocytes accumulation has deleterious effects [71].

Homocellular and heterocellular cross-talks between monocytes and endothelial cells involve multiple receptor-ligand complexes and ion channels, including gap junctions and their connexin protein building blocks, which have been compared to immunological synapses [72]. By targeting connexins and the channels they form, HSP70 may be part of the complex cascade of molecular interactions that underpin the rolling of monocytes on the endothelial wall. HSP70 interaction with TLR4, Cx43 phosphorylation and decreased expression, ATP release, and Ca^2+^ oscillations, providing several potential targets to therapeutically modulate the transendothelial migration of monocytes.

The article "Oncogenic extracellular HSP70 disrupts the gap-junctional coupling between capillary cells" was retracted in 2025. Reasons: duplicated images; original data or images not available.

**Fig 8:** Hypothetical model of the inhibitory effects of extracellular HSP70 on the diapedesis of monocytes The diagram shows the distribution of gap-junctions (double barrel) and hemichannels (single barrel) that can operate between monocytes (M) and endothelial cells of the microvascular wall. M-CSF-stimulated monocytes adhere to the endothelial cell monolayer and release HSP70 that disrupts GJIC between EC contributing to the subsequent release of ATP through Panx-1 and Cx43 hemichannels from endothelial cells. Extracellular HSP70 induce endothelial Ca^2+^ oscillations without affecting the intercellular tight junction protein, localized between apposed cells. When HSP70 is blocked (siRNA or VER155008), M-CSF-stimulated monocytes communicate with endothelial cells by gap junctions (GJIC), allowing their migration across the endothelial cell monolayer, in an endothelial Ca^2+^-dependent mechanism (slowed down by BAPTA, a Ca^2+^ chelator, Suppl. Fig. S5).

## MATERIALS AND METHODS

### Cells

Human microvascular endothelial cells (HMEC; Lonza; Basel, Switzerland) were grown in DMEM plus 10% FCS (5% CO_2_; 37°C). Human peripheral blood monocytes were isolated from buffy coats of healthy donors by Ficoll gradient (MACS system, Miltenyi Biotec Inc., Paris, Fr). CD14 monocytes isolated beads were plated in RPMI1640 plus 10% FCS and stimulated overnight by 100 ng/mL recombinant human macrophage colony-stimulating factor (M-CSF; Millipore, Molsheim, Fr). Untouched monocytes were nucleoporated with siRNA using Amaxa nucleofector kit (Amaxa; Koln, Germany) and HMEC were transfected by lipofectamine RNAiMAX (Invitrogen; Life Technologies, Saint-Aubin, Fr). siRNA HSP70 was purchased from Sigma-Aldrich (SASI_Hs01_00051449; Saint-Quentin Fallavier, Fr), siRNA Cx43 was from Santa Cruz Biotech (GJA1_human mapping 6q22.31; Clinisciences; Nanterre, Fr) and control siRNA was from Dharmacon (Fermentas; ThermoFischer, Saint-Remy-les-Chevreuses, Fr). Cells were incubated overnight in FCS-free media before use.

### Reagents

Low endotoxin rhHSP70 and rhHSP27 were purchased from Enzo Life Sciences (Villeurbanne, Fr) and rabbit anti-HSP70 from ABR (AffinityBioReagent, ThermoFisher, Fr). Mouse anti-Hsc70, rabbit anti-phospho Cx43 (Ser368, Ser255, Ser262 and Tyr265) and probenecid were from Santa Cruz Biotech. Neutralizing anti-TLR4 and mouse anti-EGFR (ErB1) were from Abcam (Cambridge, UK). Mouse anti-TLR4, polymyxin B and gefitinib were from InvivoGen (Toulouse, Fr). Rabbit anti-P-EGFR (Tyr-1068) and antiphospho- and total Akt (Ser473) were from Cell Signaling (Danvers, USA) and mouse anti-Cx43 from Invitrogen. ZO-1 antibody was from Zymed (Invitrogen). DiL-C18, thapsigargin and fura-2/AM were from Molecular Probes. VER155008 and Gap26 (VCYDKSFPISHVR) from Tocris (McKinley, USA). Other chemicals were from Sigma-Aldrich.

The article "Oncogenic extracellular HSP70 disrupts the gap-junctional coupling between capillary cells" was retracted in 2025. Reasons: duplicated images; original data or images not available.

### Specific cell treatments

To avoid endotoxin contamination of rhHSP, cells were preincubated with polymyxin B (PMB, 10 μM; 30-60 min) and rhHSP70 solutions were also treated with PMB prior to their use. To block TLR4, cells were preincubated with the neutralizing anti-hTLR4 antibody (10 μg/ml; for 30 min).

### Fluorescence recovery after photobleaching (FRAP)

The GJIC between HMEC was measured by means of gap-FRAP method [30]. Cells were loaded with 10 ng/μl of calcein/AM for 15 min. The fluorescence of investigated cells was bleached at 405 nm. The recovery of fluorescence was measured at 488 nm every 20 sec for a time period of 8 min. The fluorescence in one unbleached cell was used to correct the artefact loss of fluorescence. The permeability of gap junctions is estimated by the diffusion rate constant k (expressed in min^−1^) determined from recovery curves as following: (Fi − Ft)/(Fi – F0)=e^−kt^, where Fi, Ft and F0 are intensities before bleaching, at time t and t=0 respectively.

### Immunofluorescence and Imaging

Cells were fixed in 4% PAF and permeabilized with 0.1% Triton X-100 [31]. Images were performed using a Leica SP2 RS confocal microscope (Z-series of optical sections from 0.3-0.6 μm intervals; 512x512 pixels; Rueil-Malmaison, Fr). For co-localization, images were taken on Axio Imager 2 (Carl Zeiss GmbH) with an Apotome2 module (Optical sections of 0.5 μm; 512x512; Oberkochen, Germany).

### Triton X-100 fractionation

Triton X-100 soluble and insoluble fractions of Cx43 were separated according to VanSlyke and Musil [32]. HMEC were washed in cold PBS, scraped in PBS supplemented with N-ethylmaleide (10 mM), phenylmethylsulfonyl fluoride (1 mM), and sodium orthovanadate (1 mM), and centrifugated for 4 min at 2000g and 4°C. The pellet was resuspended in 400 μl of complete PBS plus protease inhibitor cocktail and phosphatase inhibitor cocktail 1 and 2. The suspension was incubated on ice with 1% Triton X-100 for 40 min. 175 μl of lysate was centrifugated at 100,000g for 50 min at 4°C. The supernatant was resuspended in 175 μl fractioning buffer. The remaining total lysate and the Triton X-100 insoluble fraction were sonicated for 20 s, and protein content was measured by the Bradford assay.

### Immunoprecipitation

Briefly, cells were lysed in RIPA buffer, and immunoprecipitation was performed with antibodies, as previously described [31].

### Recombinant protein production

Heat Shock 70kDa protein 1B (HSPA1B) [Homo sapiens] modified with HA Tag in Nter (rhHSP70-HA) has been produced by Proteogenix (Oberhausbergen, France). The rhHSP70 cDNA was cloned in pT7-MAT-1 expression vector in *E.coli* with His tag1 in N-terminal position (Cloning strategy: Hind III / Eco RI2). His tag is intended for affinity purification.

The article "Oncogenic extracellular HSP70 disrupts the gap-junctional coupling between capillary cells" was retracted in 2025. Reasons: duplicated images; original data or images not available.

### Cytosolic Ca^2+^ concentration

Changes in 340/380 nm ratio of Fura-2 fluorescence were used to measure [Ca^2+^]i. Briefly, cells were incubated with 2 μM fura-2-AM (40 min at 37°C), then in HEPES-buffered saline solution (HBSS) as previously described [33]. Measurements were made on Axiovert 40 (Carl Zeiss) with a 20X objective (fluor, 0.75 NA) attached to a dual-excitation spectrofluorimeter (340/380 nm). Emission (510 nm) was collected at a rate of 20 per minute.

### ATP measurement

Concentration of ATP in cell media was detected by luciferin-luciferase assay (ENLITEN ATP Assay, Promega; Charbonnieres, Fr). HMEC were plated at 500 × 10^3^ cells/cm^2^, growth arrested in FCS-free medium and exposed to apyrase (20 U/ml) or GAP26 (500 μM) or probenecid (100 μM) and/or monocytes stimulated or not by M-CSF (100 nM). Supernatants were collected after 1h to 12h, put on ice and centrifuged at 12,000 *g* for 10 min.

### Heterocellular GJIC functionality

Monocytes were labeled with 4 μM calcein/AM (30 min) together with 10 μM DiL-C18 as previously detailed [30, 34]. After washing, 10^3^ fluorescent cells were laid on HMEC monolayers. The transfer of dye was visualized after a given time at 37°C. To confirm that the calcein transfer was not due to its non-specific up-take, supernatant collected from donors were added to HMEC. No dye uptake by HMEC was found within 24h.

### HSP70 ELISA analyses

HSP70 levels in cell supernatants were evaluated using enzyme-linked immunoabsorbent assay (ELISA kit; Enzo Life Sci. ADI-EKS-715) according to the protocol provided.

### Transendothelial cell migration

HMEC were cultured on 3-μm membrane pores of Transwell inserts until confluency, then FCS-free overnight (CytoSelectTM, Cell Biolabs; Euromedex, Mundolsheim, Fr). 300 μl of monocytes suspension were added (3×10^5^ cells per well). After 3-hours, migrated cells were labeled with phycoerythrin-conjugated anti-CD14+ antibody and counted by flow cytometry.

### Statistical analysis

One-way analysis of variance (ANOVA; Statview Software) was used to compare data groups of at least five independent experiments. Stimulated samples were compared to controls by two-tailed, unpaired t-tests. *P values < 0.05 were significant.

## SUPPLEMENTARY MATERIALS AND FIGURES


